The article "Research on the Relationship between Urban Agricultural Nonpoint Source Pollution and Rural Residents' Income Growth" was published in 2022. Journal: J Environ Public Health.

# Research on the Relationship between Urban Agricultural Nonpoint Source Pollution and Rural Residents' Income Growth

**DOI:** 10.1155/2022/4133245

**Published:** 2022-08-10

**Authors:** Pu Xu, Shanwei Li, Xiaona Yang, Yufeng Li

**Affiliations:** School of Economics and Management, Shanghai Ocean University, Shanghai 201306, China

## Abstract

Researching the relationship between urban agricultural nonpoint source pollution (*UANSP*) and increases in rural residents' income levels has significant practical implications for effectively controlling *UANSP* and improving the quality of life of urban residents, and it is conducive to achieving a win-win situation between economic and environmental benefits. This study chooses agricultural statistical data from Shanghai from 1998 to 2019, implements the *EKC* and the *VAR* model to dynamically analyze internal interaction between them, and thoroughly examines impact effect and explanatory contribution degree of each variable. The results show the following: (1) There was an inverted “*N*” curve between plastic film application intensity and rural residents' per capita disposable income; there was a linear decreasing relationship between the intensity of fertilizer and pesticide application and rural residents' per capita disposable income. (2) Nonpoint source pollution emissions will decrease as rural residents' income levels rise. Reduction of nonpoint source pollution can promote the short-term improvement of rural residents' income levels, but it has a negative effect on the long-term improvement of rural residents' income levels. (3) Fertilizer and pesticide application intensity had a low driving effect on rural residents' income growth, whereas plastic film application intensity had a strong driving effect. Therefore, the *ANSP* of Shanghai should be treated from both long-term and short-term perspectives on the basis of decreasing stage. In the long term, the government should increase farmers' sense of ownership in agricultural nonpoint source pollution control, prioritize the development of ecological circular agriculture, and gradually improve nonpoint source remote sensing monitoring and service management capabilities. In the short term, the government should reduce farmers' nonpoint source pollution through subsidies and technical assistance. To keep costs down, the government established an administrative reward and punishment system to control *ANSP* at the source.

## 1. Introduction

Urban agriculture is the “pioneer” of modern agricultural development. Urban agriculture is different from ordinary agricultural areas in a number of respects. On the one hand, the urban area's limited agricultural resources necessitate the provision of a huge supply of agricultural products to its citizens. On the other hand, agricultural nonpoint source pollution (*ANSP*) caused by excessive agricultural resource usage endangers the urban living environment [1–4]. Fertilizer; pesticide residues; agricultural films widely used throughout agriculture; and agrarian or rural wastes such as crop residues, animal urine, manure, domestic sewage, and garbage are really the major causes of *ANSP*. It exhibits inconsistencies in its emission properties, making it difficult to identify and monitor [5–7]. *ANSP* not only jeopardizes local agricultural and drinking water, but also contaminates soil and surface water [8, 9]. In China, the intensive input of production elements is critical to China's agricultural development. Agriculture under the concentrated management model is characterized by high yield, low efficiency, and high input [6, 10]. While such an extensive production strategy helps agricultural economic growth, it also threatens to undermine the agroecological ecosystem [11, 12]. In agricultural production, the *ANSP* generated by agricultural chemicals like fertilizer, pesticide, and plastic films, in particular, has become a detrimental factor that endangers the water and soil environment [13, 14]. The shortage of agricultural resources has become more and more evident in cities, and agriculture will become indispensable to cities and their citizens. It has progressed from maintaining the supply of agricultural products to performing a variety of complex functions, and from auxiliary duties to core functions. Prevention and control of *ANSP* are linked to the investment environment, urban construction, urban image, quality of life, ecological balance, tourism, culture, and other factors and will ultimately affect the city's overall competitiveness [15, 16]. As a result, efficient control of urban agricultural nonpoint source pollution (*UANSP*) is a critical component of ecological environmental protection and the key to fostering the long-term development of urban agriculture, which is conducive to achieving a win-win situation in terms of economic and environmental benefits [17–20].

The article "Research on the Relationship between Urban Agricultural Nonpoint Source Pollution and Rural Residents' Income Growth" was published in 2022. Journal: J Environ Public Health.

According to the Environmental Kuznets Curve (*EKC*) hypothesis, the relationship between environmental pollution and economic growth is an inverted “*U*” shape, which implies that environmental quality begins to deteriorate with economic growth and gradually improves after a certain level of economic growth is attained [21–24]. People have long been concerned about the conflict between agricultural economic development and environmental protection. At present, there is no consensus on whether the *EKC* hypothesis exists in *ANSP* in different countries and regions [25]. In terms of China studies, Hui used the *EKC* to investigate the link between *ANSP* and income in 30 provinces and cities in China. According to his research, the relationship between the two is shaped like an inverted “*U*,” which is consistent with the *EKC* hypothesis [26]. In terms of American studies, through the *EKC* hypothesis, Managi empirically analyzed the relationship between economic growth and mitigation of environmental degradation using agricultural data from 48 states in the United States. The findings indicate that lowering pesticide contamination promotes agricultural economic growth [27]. In relation to specific pollutant indicators, the agricultural economy and environmental pollution continue to exhibit “*N*” type, inverted “*N*” type, or linear change characteristics [28]. Liu et al. used the *EKC* to examine chemical fertilizer applications in China from 1978 to 2017, with Hubei Province as a case study. The findings revealed that the growth of farmers' income and the use of chemical fertilizer followed an “*N*” shaped pattern [29]. It can be found that there are variances in the relationship between *ANSP* and agricultural economic growth that do not fully conform to the *EKC* hypothesis. Furthermore, on the one hand, the *EKC* hypothesis ignores the two-way influence mechanism and dynamic correlation effect between *ANSP* and agricultural economic growth, raising the possibility of variable endogeneity bias [30]. On the other hand, most existing research focuses on conventional agricultural areas, and there is still a scarcity of studies on the relationship between *ANSP* and agricultural economic growth from an urban perspective. For this reason, researching the relationship between *UANSP* and agricultural economic growth has substantial practical significance for effectively reducing environmental pollution and increasing the quality of life for urban residents.

Shanghai, as an international metropolis, has evident regional specificity and significant advantages in terms of location, technology, talent, market, and money, despite the scarcity of agricultural and environmental resources. Shanghai's agriculture not only plays a vital role in utilizing nearby villages to adjust the climate, purify the air, mitigate the urban “heat island effect,” and improve the ecological environment of megacities, but also provides strategic space for the city's core functions and undertakes more diverse and high-level energy levels of economic development functions. Therefore, this study uses Shanghai as the research object for *UANSP* and develops an *EKC* model between the application intensity of fertilizers, pesticides, and plastic film and rural residents' per capita discretionary income, as well as describing the morphological relationship and trend characteristics of each variable. Based on the research on the evolution characteristics of *ANSP* and economic growth in Shanghai, the dynamic impact effect and interaction mechanism between *ANSP* and per capita disposable income of rural residents were investigated using the impulse response function and variance decomposition method from a time series perspective. This study is expected to serve as an example for the development of *UANSP* prevention and control policies in Shanghai and other cities.

The article "Research on the Relationship between Urban Agricultural Nonpoint Source Pollution and Rural Residents' Income Growth" was published in 2022. Journal: J Environ Public Health.

## 2. Material and Methods

### 2.1. Data Sources

We take Shanghai as an example; the scale of planting in Shanghai's agricultural production is large, the scale of breeding is small, and the agricultural resources consumed are primarily fertilizer, pesticide, and plastic films. Three indicators of fertilizer application intensity (*NPK*, kg/hm^2^), pesticide application intensity (*Pestic*, kg/hm^2^), and plastic film application intensity (*PF*, kg/hm^2^) were chosen as the Shanghai's *ANSP* index based on agricultural production characteristics. Based on 1998 data, this research chooses rural residents' per capita disposable income as an indicator of agricultural economic progress. The following indicators are derived from the amount of fertilizers applied, the amount of pesticide applied, the effective irrigation area, the amount of plastic film applied, and the area covered by plastic film. The following is the computation method:

Fertilizer application intensity (kg/hm^2^) = amount of fertilizers applied/effective irrigation area.

Pesticide application intensity (kg/hm^2^) = amount of pesticide applied/effective irrigation area.

Plastic film application intensity (kg/hm^2^) = amount of plastic film applied/plastic film coverage area.

Data from 1998 to 2019 were obtained from “China Environmental Statistical Yearbook,” “China Agricultural Yearbook,” “China Agricultural Statistics,” “Shanghai National Economic and Social Development Historical Statistics,” and “Shanghai Statistical Yearbook.”

### 2.2. Model Method

#### 2.2.1. *EKC* Analysis

(1) $$\begin{array}{c} Y_{i}=\beta_{0}+\beta_{1}M+\beta_{2}M^{2}+\beta_{3}M^{3}+\varepsilon , \end{array}$$

where *Y*_*i*_ is indeed the *ANSP* index (*i* = *NPK*, *Pestic*, *PF*); *M* is rural residents' per capita disposable income; *n* (*n* = 0, 1, 2, 3) is the regression coefficient, whose coefficient symbol determines the shape of the *EKC*; and *ε* is the random disturbance term. The various values of model coefficients *β*_0_, *β*_1_, *β*_2_, and *β*_3_ reflect the various relationships between *ANSP* and per capita disposable income of rural residents (as shown in Table 1).

The article "Research on the Relationship between Urban Agricultural Nonpoint Source Pollution and Rural Residents' Income Growth" was published in 2022. Journal: J Environ Public Health.

#### 2.2.2. *VAR* Model

The *VAR* (vector autoregression) model is a widely known econometric model for analyzing time series as it can describe the linear relationship between variables in the same sample period as their past values. The formula is as follows:

(2) $$\begin{array}{c} Y_{i}=A_{1}Y_{i-1}+A_{2}Y_{i-2}+\ldots A_{p}Y_{i-p}+\delta_{i};t=1,2,\ldots ,T, \end{array}$$

where *Y*_*t*_ represents time series vector, *A*_*p*_ represents time series coefficient matrix, *P* represents order of autoregressive lag, and *δ*_*t*_ represents error vector.

#### 2.2.3. Impulse Response Function and Variance Decomposition

Because a single regression coefficient has a large impact on results, the *VAR* model uses impulse response function and variance decomposition to analyze the dynamic impact effect between variables as well as the explanatory contribution degree on the whole. Impulse response function is used to analyze response change and response direction of a random error term in a model after it has been impacted by one standard deviation. The formula is as follows:

(3) $$\begin{array}{c} y_{i}=\alpha +\varphi_{0}\varepsilon_{i}+\varphi_{1}\varepsilon_{i-1}+\varphi_{2}\varepsilon_{i-2}+\cdots =\alpha +\sum_{j=0}^{\infty }\varphi_{j}\varepsilon_{i-j}\text{,}\\ \frac{\partial y_{i+s}}{\partial \varepsilon_{i}}=\varphi_{s}. \end{array}$$

Variance decomposition is another method to measure the *VAR* model, which depicts the contribution rate of each endogenous variable in model to system variable in order to assess relative importance of impulse disturbance term to the model variable. The formula is as follows:

(4) $$\begin{array}{c} y_{i+h}-{\hat{y}}_{i+h}=\varphi_{0}\varepsilon_{i+h-1}+\cdots +\varphi_{h-1}\varepsilon_{i+1}=\sum_{i=0}^{h-1}\varphi_{i}\varepsilon_{i+h-i}\text{,}\\ y_{i+h}-{\hat{y}}_{i+h}=\sum_{i=0}^{h-1}\varphi_{i}\varepsilon_{i+h-i}=\sum_{i=0}^{h-1}\varphi_{i}PP^{-1}\varepsilon_{i+h-i}=\sum_{i=0}^{h-1}\omega_{i}\nu_{i+h-i}\text{,} \end{array}$$

where *v*_*i*_ _*+*_ _*h-i*_ represents the orthogonalization shock. The contribution of the first variable's dynamic action to *y*_*j,i*_ _*+*_ _*h*_ prediction error is calculated further as follows:

(5) $$\begin{array}{c} \frac{\omega_{0,j1}^{2}+\cdots +\omega_{h-1,j1}^{2}}{\sum_{k=1}^{n}\omega_{0,jk}^{2}+\cdots +\omega_{h-1,jk}^{2}}. \end{array}$$

Formula (5) calculates the contribution ratio as a function of the prediction period *h*, and the sum of the contribution ratios of all variables to the prediction error is 1.

The article "Research on the Relationship between Urban Agricultural Nonpoint Source Pollution and Rural Residents' Income Growth" was published in 2022. Journal: J Environ Public Health.

## 3. Evolutionary Characteristics of Economic Growth of *ANSP*

*EKC* tests were conducted on plastic film, chemical fertilizer, pesticide, and per capita disposable income of rural residents, according to the *EKC*. When the curve fitting results of the quadratic and cubic equations were compared, it was discovered that the cubic equation had the best curve fitting effect, so the cubic equation's curve fitting results were chosen, as shown in Table 2 and Figure 1.

Based on the *EKC* results of plastic film application intensity and per capita disposable income of rural residents, the fitting curve's Sig value was 0.001 < 0.01, and *R*^2^ = 0.575. As can be seen, the cubic curve fits well and can be investigated further. According to the research results, the relationship between plastic film application intensity and rural residents' per capita disposable income appears to follow an inverted “*N*” curve. It demonstrates that as rural residents' disposable income increases, plastic film application intensity in agriculture undergoes a “decline⟶rise⟶decline” change process, with two inflection points in the inverted “*N*” curve. According to the derivation of the unary cubic equation function, the application intensity of plastic film corresponding to the inflection point of the *EKC* principle is 217.89 kg/hm^2^ and 273.63 kg/hm^2^ for the per capita disposable income of rural residents. According to data, the per capita disposable income of Shanghai's rural residents crossed the first turning point in 2011. In 2017, rural residents' per capita incomes did pass the second turning point. By 2019, the per capita disposable income of rural residents in Shanghai had been to the right of the second inflection point, and plastic film application intensity had been decreasing. This demonstrates that as rural residents' income levels rise in Shanghai, so does their quality of life, which does have a positive impact on the reduction of agricultural plastic film pollution.

Based on the *EKC* results of fertilizer application intensity and per capita disposable income of rural residents, the fitting curve's Sig value was 0.001 < 0.01, and *R*^2^ = 0.778. As can be seen, the cubic curve fits well and can be investigated further. According to the research results, there was a decreasing linear relationship between fertilizer application intensity and rural residents' per capita disposable income. In terms of rural residents' levels of income, fertilizer application intensity has been shrinking since 1998, as per capita disposable income has increased, and the downward trend has gradually accelerated.

Based on the *EKC* results of pesticide application intensity and per capita disposable income of rural residents, the fitting curve's Sig value was 0.001 < 0.01, and *R*^2^ = 0.741. As can be seen, the cubic curve fits well and can be investigated further. According to the research results, there was a decreasing linear relationship between pesticide application intensity and rural residents' per capita disposable income. It demonstrates that, since 1998, with the dramatic rise in rural residents' levels of income, the pesticide application intensity in Shanghai has shown a downward trend. According to the fitting curve, the rate of decrease in pesticide application intensity in Shanghai slowed from 2008 to 2012, but after 2013, the pesticide application intensity has shown a rapid downward trend, which is likely to be related to China's establishment of a fully grown *ANSP* prevention and control policy system [31].

The article "Research on the Relationship between Urban Agricultural Nonpoint Source Pollution and Rural Residents' Income Growth" was published in 2022. Journal: J Environ Public Health.

Finally, the relationship between plastic film application intensity and rural residents' per capita disposable income in Shanghai is shaped like an inverted “*N*,” and the *EKC* theory inflection point was crossed in 2011 and 2017. Prior to 2010, Shanghai's cultivated land area decreased year after year, resulting in a decrease in mulching film application intensity and the first inflection point. The mulching film application intensity in Shanghai has been fluctuating at 246 kg/hm^2^ since 2010, and the second inflection point appeared as the Shanghai government increased its efforts to manage the human settlement environment. Fertilizer application intensity, plastic film application intensity, and rural resident per capita disposable income decreased. The reason for this is that the arable land area in Shanghai has been decreasing year by year, and the upgrading of agricultural product consumption demand has resulted in a significant decrease in the use of fertilizer and pesticide in agricultural production by rural residents. As a result, it is necessary to master the current situation of the use of chemical fertilizers, pesticides, and mulching film in Shanghai and determine whether their application effects hinder farmers' economic income and lead to agricultural nonpoint source pollution, which needs to be discussed further from other perspectives.

## 4. Economic Driving Characteristics of *ANSP*

The *EKC* can explicitly explore form and trend characteristics between *ANSP* in Shanghai and rural residents' income levels and can determine whether there is an inflection point in *ANSP* when rural residents' income level increases, but the curve fails to provide in-depth proof of the inherent logical relationship and dynamic influence between the two, and the *VAR* model can compensate for the *EKC* model's limitations. The model can analyze the dynamic effects of random disturbances on endogenous variables by using *ANSP* and per capita disposable income of rural residents as system endogenous variables. As a result, this paper employs the *VAR* model to conduct an empirical analysis of *ANSP* and rural resident income level in Shanghai, dynamically analyzes the internal interaction between the two, deeply discusses the impact effect, and explains the contribution of each variable.

The article "Research on the Relationship between Urban Agricultural Nonpoint Source Pollution and Rural Residents' Income Growth" was published in 2022. Journal: J Environ Public Health.

### 4.1. Stability Check

1. *ADF* test. During the process of developing the *VAR* model, to avoid the pseudo-regression phenomenon during the time series analysis process, the data should really be tested for stationarity. *ADF* unit root test is used in this paper to perform the stationarity test. When the *ADF* test value of each variable is less than the 5% horizontal critical value, it means that the variable belongs to a stationary series; otherwise, it belongs to a nonstationary series. Concurrently, to eliminate potential influence of heteroscedasticity in data, logarithms within each variable were used to ensure model's stability. The findings of unit root test of *LnNPK*, *LnPestic*, *LnPF*, and *LnFarm* (as shown in Table 3) show that only *LnFarm* is a nonstationary sequence in the original variables, but after the first-order difference, *ADF* values of all variables are less than 5% significant, which meets *VAR* modeling requirements.
2. Lag order determination and *VAR* model results. To ensure the model's validity, the lag period should be evaluated when constructing a *VAR* model. The lag order of the *VAR* model constructed by agricultural nonpoint source pollution and rural residents' income level is 1 based on AIC and SC information values in Table 4. Each variable is applied to first-order lag vector autoregression as a consequence. After regression, the goodness of fit is greater than 0.9, indicating that the model is reasonable and can accurately reflect the dynamic relationship between variables.

### 4.2. Johansen Co-Integration Test

The Johansen co-integration test method is used in this paper to test *LnNPK*, *LnPestic*, *LnPF*, and *LnFarm* variables to ascertain whether there is any long-term stable co-integration relationship between many variables (as shown in Table 5). The findings demonstrate that *VAR* model rejects null hypothesis of “no co-integration relationship” at a 5% level of significance, and there are two co-integration relationships in the model, implying a long-term stable co-integration relationship between the variables. As a result, impulse response function and variance decomposition method can be used for additional analysis to scrutinize dynamic relationship and synergistic mechanism between growth of rural residents' per capita disposable income and plastic film, fertilizers, and pesticide.

The article "Research on the Relationship between Urban Agricultural Nonpoint Source Pollution and Rural Residents' Income Growth" was published in 2022. Journal: J Environ Public Health.

### 4.3. Impulse Response Analysis

To research dynamic effects of plastic film, fertilizer, pesticide application intensity, and rural residents' per capita discretionary income, an impulse response function model was developed to explain the degree of impact between various endogenous variables, and an impulse response graph was created [32]. The horizontal axis represents the lag period, while the vertical axis represents the response degree.

Figure 2(a) demonstrates that per capita disposable income of rural residents adds one standard error shock disruption to plastic film application intensity. The impulse response value of the first to fifteenth period varies within the range of [−0.0185, 0], and the average driving effect of the first to fifteenth period is −0.0148. The negative inhibitory effect of rural residents' per capita disposable income on plastic film application intensity gradually increased from the first to fifth period, and the overall inhibitory effect from the sixth to fifteenth period showed a gentle trend. It has been shown that the negative impact of rural residents' per capita disposable income on plastic film application intensity has a rising trend and then shrinks. This illustrates that as time passes, the per capita disposable income of rural residents has an inhibitory effect on the application strength of plastic films, and this inhibitory effect tends to increase initially before stabilizing.  Figure 2(b) demonstrates that plastic film application intensity adds one standard error shock disruption to rural residents' per capita disposable income, and impulse response value from the first to fifteenth period fluctuates within the range of [−0.0122, 0.0028]. From the first to the third period, plastic film application intensity has a significant inhibitory effect on rural residents' per capita disposable income, with an average driving effect of −0.0064. It exhibited a positive promotion effect after the fourth to eleventh periods, while the impulse response amplitude of the twelfth to fifteenth periods decreased noticeably and showed an inhibitory effect, eventually approaching −0.0009 smoothly. This illustrates that, in the short term, the effect of plastic film application intensity on per capita disposable income of rural residents exhibits an “inhibition⟶promotion⟶inhibition” trend. In the long term, the overall impulse response is found to have a negative inhibitory effect, but the effect is quite tiny.

The article "Research on the Relationship between Urban Agricultural Nonpoint Source Pollution and Rural Residents' Income Growth" was published in 2022. Journal: J Environ Public Health.

Figure 2(c) demonstrates that per capita disposable income of rural residents adds one standard error shock disruption to fertilizer application intensity. The impulse response value of the first to fifteenth period varies within the range of [−0.0099, 0], and the average driving effect of the first to fifteenth period is −0.0075. The negative inhibitory effect of rural residents' per capita disposable income on fertilizer application intensity gradually increased from the first to sixth period, and the overall inhibitory effect from the seventh to fifteenth period showed a gentle trend. On the whole, the effect of rural residents' per capita disposable income on the fertilizer application intensity reveals that the inhibitory effect rises and then stabilizes over time.  Figure 2(d) demonstrates that fertilizer application intensity adds one standard error shock disruption to rural residents' per capita disposable income, and impulse response value from the first to fifteenth period fluctuates within the range of [−0.0065, 0.0107]. From the first to the fourth period, fertilizer application intensity has a significant positive effect on rural residents' per capita disposable income, with an average driving effect of 0.0058. The average driving effect is −0.0052, and the overall income has a negative inhibitory effect. It has been shown that overall impact of fertilizer application intensity on rural residents' per capita disposable income is a promotion effect in initial stages and an inhibitory effect in the subsequent stages, which means the income rises first and then gradually stabilizes.

Figure 2(e) demonstrates that rural residents' per capita disposable income adds one standard error shock disturbance to pesticide application intensity, impulse response value of the first period is 0, and impulse response value of the second to fifteenth periods is in the range of [−0.0113, 0.0006]. Among them, rural residents' per capita disposable income in the second period has a significant positive promotion effect on the intensity of pesticide application, with an impulse response value of 0.0006. From the third to fifteenth period, rural residents' per capita disposable income had a negative inhibitory effect on pesticide application intensity, with an average driving effect of −0.0081. From the third to eighth periods, rural residents' per capita disposable income had a significant negative inhibition effect on pesticide application intensity, and impact intensity increased gradually. As a whole, inhibition effect indicates a smooth trend from the ninth to fifteenth periods, eventually stabilizing at −0.0112. Overall, effect of rural residents' per capita disposable income on pesticide application intensity is generally a facilitation effect in the beginning period and an inhibitory effect that increases first and then gradually stabilizes in the later phase.  Figure 2(f) demonstrates that pesticide application intensity adds one standard error shock disruption to rural residents' per capita disposable income, and impulse response value from the first to fifteenth period fluctuates within the range of [−0.0137, 0.0236]. From the first to the fourth period, pesticide application intensity has a significant positive effect on rural residents' per capita disposable income, with an average driving effect of 0.0146. The average driving effect is −0.0108, and overall income has a negative inhibitory effect. It has been shown that overall impact of pesticide application intensity on rural residents' per capita disposable income is a decreasing promotion effect in initial stages and an inhibitory effect in the subsequent period, which raises first and then gradually stabilizes.

The article "Research on the Relationship between Urban Agricultural Nonpoint Source Pollution and Rural Residents' Income Growth" was published in 2022. Journal: J Environ Public Health.

To summarize, the impact of *LnFarm* on *LnPF*, *LnNPK*, and *LnPestic* can be seen in the above three groups of impulse response functions as an inhibitory effect that increases initially and then gradually stabilizes. The effect of *LnNPK* and *LnPestic* on *LnFarm* revealed that first to fourth periods had a decreasing promotion effect and fifth to fifteenth periods had an inhibitory effect that increased initially and then gradually stabilized. The influence of *LnPF* on *LnFarm* revealed a fluctuating inhibitory effect. As a whole, the amount of *ANSP* in Shanghai will decrease as rural residents' income levels rise. Nonpoint source pollution reduction can improve rural residents' income in the short term, but it is not conducive to rural residents' income growth in the long run. The reason for this could be that, as shown in Figure 1, the application intensity of the *ANSP* index is relatively stable in the short term, and the input of plastic film, fertilizer, and pesticide can increase rural residents' income and promote agricultural economic growth to a degree. That is, in the threshold range, a short-term increase in agricultural inputs is beneficial to increasing the income of rural residents. Long-term films and the use of fertilizers and pesticides accumulate for farmers and unreasonable fertilization on farmland. In this instance, the long-term accumulation of agricultural pollution is challenging to address in a timely manner, impacting the output of agricultural products, and it is demonstrated as the inhibiting effect of ANSP on the rise in the income level of rural inhabitants. That is, the long-term use of agricultural inputs is detrimental to the income of rural residents. To achieve stable income growth for rural residents, it is necessary to comprehensively measure long-term and short-term benefits, to continuously reduce *ANSP* emissions on the one hand and to reduce the negative effects of *ANSP* on the agricultural environment on the other hand.

The article "Research on the Relationship between Urban Agricultural Nonpoint Source Pollution and Rural Residents' Income Growth" was published in 2022. Journal: J Environ Public Health.

### 4.4. Variance Decomposition

Variance decomposition can decompose variance of a variable in a *VAR* model system into various disturbance terms and assess degree of influence of their interaction. This paper employs the variance decomposition method to investigate the interpretive significance and importance of each index of *ANSP* in Shanghai to the growth of rural residents' per capita disposable income, in addition to analyzing the contribution of each systemic shock to the change of endogenous variables. According to Table 6, in the decomposition of rural residents' disposable income, the average contribution of mulching film application intensity, fertilizer application intensity, and pesticide application intensity changes to the growth of rural residents' income level is 28.44 percent, 5.82 percent, and 4.34 percent, respectively. The results also showed that fertilizer and pesticide application intensity had a minor impact on the increase in rural residents' income, whereas plastic film application intensity had a significant impact. Simultaneously, average self-contribution degree of rural residents' income growth is 61.40 percent, which is average self-contribution rate after excluding plastic film, fertilizer, and pesticide emissions, and primarily includes agricultural mechanization level, production and operation mode, number of agricultural employees, and agricultural technology application and comprehensive development.

## 5. Conclusion and Suggestions

### 5.1. Conclusion

Academic researchers have long focused on the interaction between agricultural nonpoint source pollution and agricultural economy. This paper employs time series data to investigate dynamic relationship between *ANSP* and income level of rural inhabitants in Shanghai. According to the results of the *EKC* analysis, its intensity of mulching film application in Shanghai does have an inverted “*N*” curve relationship to rural residents' per capita disposable income. There was a diminishing linear association between the intensity of fertilizer and pesticide application and rural residents' per capita disposable income. Shanghai is currently on the right side of the *EKC*, and the intensity of plastic film, fertilizer, and pesticide applications will continue to decline and stabilize. A *VAR* model was used to examine the dynamic relationship and mechanism between *ANSP* and the income level of rural residents in Shanghai. The application intensity of plastic film, fertilizer and pesticide, and the per capita disposable income of rural residents showed inhibitory effect on each other. According to variance decomposition results, application intensity of fertilizer and pesticides had a little driving impact on the growth in rural residents' income, but application intensity of plastic film had a more noticeable driving effect. This reveals that agricultural contamination induced by the use of fertilizers and pesticides is not immediately apparent. In comparison to fertilizers and pesticides, rural residents' desire for plastic film increases as their economic level rises. Plastic film overuse is a significant *ANSP* concern in Shanghai. Although *ANSP* is reducing in Shanghai, the long-term unreasonable and excessive use of chemical inputs such as plastic film, fertilizer, and pesticide continues to have negative effects on the agricultural environment, and the problem of *ANSP* cannot be solved naturally in the short term.

The article "Research on the Relationship between Urban Agricultural Nonpoint Source Pollution and Rural Residents' Income Growth" was published in 2022. Journal: J Environ Public Health.

### 5.2. Suggestions

According to the findings of the preceding studies, economic development will result in the generation of agricultural nonpoint source pollution, as many scholars have concluded [33–35]. This paper demonstrates, through empirical research, that *ANSP* in Shanghai has entered a period of decline, and an improvement trend in Shanghai's agricultural environment is forming. To maintain this trend, not only should environmental governance policies and measures be strictly implemented, but more active ecological protection actions should be taken as well. On this basis, the best strategy for reducing *ANSP* while maintaining long-term economic growth for rural residents can be a composite of long-term and short-term considerations.

In the long term, the government encourages farmers to actively respond to the call, recognize the importance of *ANSP* control, establish farmland protection and nonpoint source pollution control subject consciousness, and improve their awareness of environmental protection and social responsibility sharing. On the other hand, the government should promote agricultural input reduction, clean production, waste recycling, and an ecological industry model, and the priority should be given to the development of an ecological circular agriculture mode for producers to provide green technology, increase capital and technology for nonpoint source remote sensing monitoring, and gradually improve the level of nonpoint source remote sensing monitoring and service management capabilities.

In the short term, the government should, on the one hand, gain a better understanding of farmers' willingness to participate in *ANSP* control and the factors that affect it, reduce farmers' nonpoint source pollution control costs through subsidies and technical assistance, and relieve farmers' financial stress. On the other hand, the government should use managerial means to establish reward and punishment mechanisms, orderly guide farmers to improve plastic film recovery rates and motivate the use of degradable plastic film and other new materials, strengthen the promotion of green fertilizer and organic fertilizer, establish a centralized pesticide distribution system, and control *ANSP* at the source.

The article "Research on the Relationship between Urban Agricultural Nonpoint Source Pollution and Rural Residents' Income Growth" was published in 2022. Journal: J Environ Public Health.

Shanghai is used as an example in this paper, and the selection of indicators is based on the current situation of the region, which may lead to the limitations of the research results. In view of the limited academic ability of this paper, there may be differences in the selection of research objects, and the thinking on the problem is not mature enough. It is expected that relevant scholars can supplement and improve the study on urban agricultural nonpoint source pollution in follow-up research, so as to promote the sustainable development of urban agriculture.

## Figures and Tables

**Figure 1:** Fitting curve of the *ANSP* index and rural residents' per capita disposable income.

**Figure 2:** Impulse response graph between the application intensity of *NPK*, pesticides, and plastic film and economic growth. (a) Response of *LnFarm* to *LnPF*. (b) Response of *LnPF* to *LnFarm*. (c) Response of *LnFarm* to *LnNPK*. (d) Response of *LnNPK* to *LnFarm*. (e) Response of *LnFarm* to *LnPestic*. (f) Response of *LnPestic* to *LnFarm*.

**Table 1:** Relationship between *ANSP* and per capita disposable income of rural residents.

Value of coefficients	Variable relationship
*β *_1_ > 0, *β*_2_ = 0, *β*_3_ = 0	A simple increasing linear relationship
*β *_1_ < 0, *β*_2_ = 0, *β*_3_ = 0	A simple decreasing linear relationship
*β *_1_<0, *β*_2_>0, *β*_3_ = 0	A positive “*U*” curve relationship
*β *_1_ > 0, *β*_2_ < 0, *β*_3_ = 0	An inverted “*U*” curve relationship
*β *_1_ > 0, *β*_2_<0, *β*_3_>0	A positive “*N*” curve relationship
*β *_1_<0, *β*_2_>0, *β*_3_ < 0	An inverted “*N*” curve relationship
*β *_1_ = 0, *β*_2_ = 0, *β*_3_ = 0	No linear relationship

**Table 2:** Comparison of curve fitting effects.

Variables	Goodness of fit (*R*^2^)	
	Quadratic equation fitting	Cubic equation fitting
*PF*	0.393	0.575
*NPK*	0.778	0.778
*Pestic*	0.740	0.741

**Table 3:** Influencing factor index stationarity test.

Sequences	(C, T, K)	ADF statistics	0.05 critical value	Conclusion
*LnNPK*	(C, T, 0)	−4.1602	−3.6450	Stationary
*LnPestic*	(0, 0, 0)	−2.4708	−1.9581	Stationary
*LnPF*	(C, 0, 0)	−6.3853	−3.0124	Stationary
*LnFarm*	(C, T, 0)	−3.6233	−3.6584	Nonstationary
*DLnNPK*	(C, T, 0)	−10.392	−3.6584	Stationary
*DLnPestic*	(C, 0, 0)	−4.6850	−3.0207	Stationary
*DLnPF*	(0, 0, 0)	−4.6566	−1.9591	Stationary
*DLnFarm*	(C, 0, 1)	−3.6091	−3.0299	Stationary

*Note.* In (C, T, K), C means intercept, T means trend, K means lag, and 0 means no intercept or trend.

The article "Research on the Relationship between Urban Agricultural Nonpoint Source Pollution and Rural Residents' Income Growth" was published in 2022. Journal: J Environ Public Health.

**Table 4:** Model lag order.

Lag	AIC	SC
0	−3.8491	−3.6502
1	−13.0959^∗^	−12.1011^∗^

Note: ^∗^Represents the optimal lag order.

**Table 5:** Johansen co-integration test.

Hypothesized No. of CE(s)	Eigenvalue	Trace test		Maximum eigenvalue	
		Trace statistic	0.05 critical value	Max-eigen statistic	0.05 critical value
None^∗^	0.9168	84.2646	47.8561	52.2053	27.5843
At most 1^∗^	0.6714	32.0593	29.7971	23.3685	21.1316
At most 2	0.3365	8.6909	15.4947	8.6148	14.2646
At most 3	0.0036	0.0761	3.8415	0.0761	3.8415

*Note.* ^∗^denotes rejection of the hypothesis at the 0.05 level.

**Table 6:** Variance decomposition table of disposable income of rural residents.

Period	SE	*LnFarm*	*LnPF*	*LnNPK*	*LnPestic*
1	0.0171	100	0	0	0
2	0.0261	93.0320	6.5933	0.3303	0.0445
3	0.0345	83.5210	15.2402	1.2103	0.0284
4	0.0425	74.7705	22.6352	2.3908	0.2036
5	0.0501	67.5611	28.0596	3.6460	0.7333
6	0.0572	61.8488	31.7078	4.8387	1.6047
7	0.0637	57.3920	33.9962	5.8997	2.7122
8	0.0697	53.9389	35.3268	6.8043	3.9301
9	0.0752	51.2735	36.0216	7.5540	5.1510
10	0.0802	49.2208	36.3162	8.1636	6.2995
11	0.0848	47.6412	36.3734	8.6536	7.3318
12	0.0892	46.4243	36.3004	9.0455	8.2298
13	0.0932	45.4828	36.1652	9.3588	8.9932
14	0.0971	44.7482	36.0089	9.6104	9.6325
15	0.1008	44.1671	35.8547	9.8145	10.1637
Mean	0.0654	61.4015	28.4400	5.8214	4.3372

## Data Availability

Data from 1998 to 2019 were obtained from “China Environmental Statistical Yearbook,” “China Agricultural Yearbook,” “China Agricultural Statistics,” “Shanghai National Economic and Social Development Historical Statistics,” and “Shanghai Statistical Yearbook.” All data included in this study can be obtained from the corresponding author upon request.

## References

[1] Ayub R., Messier K. P., Serre M. L., Mahinthakumar K. (2019). Non-point source evaluation of groundwater nitrate contamination from agriculture under geologic uncertainty. *Stochastic Environmental Research and Risk Assessment*.

[2] Opitz I., Berges R., Piorr A., Krikser T. (2016). Contributing to food security in urban areas: differences between urban agriculture and peri-urban agriculture in the Global North. *Agriculture and Human Values*.

[3] Zhou Y., Han J., Li J., Zhou Y., Wang K., Huang Y. (2021). Building resilient cities with stringent pollution controls: a case study of robust planning of Shenzhen City’s urban agriculture system. *Journal of Cleaner Production*.

The article "Research on the Relationship between Urban Agricultural Nonpoint Source Pollution and Rural Residents' Income Growth" was published in 2022. Journal: J Environ Public Health.

[4] Liu Z., Lang L., Hu B., Shi L., Huang B., Zhao Y. (2021). Emission reduction decision of agricultural supply chain considering carbon tax and investment cooperation. *Journal of Cleaner Production*.

[5] Jiang Z. y., Hu Y. (2021). Coupling and coordination between new urbanization and agricultural modernization in Central China. *Journal of Natural Resources*.

[6] Withers P. J., Neal C., Jarvie H. P., Doody D. (2014). Agriculture and eutrophication: where do we go from here?. *Sustainability*.

[7] Tang Z., Engel B. A., Pijanowski B. C., Lim K. (2005). Forecasting land use change and its environmental impact at a watershed scale. *Journal of Environmental Management*.

[8] Huang L., Ban J., Han Y. T., Yang J., Bi J. (2013). Multi-angle indicators system of non-point pollution source assessment in rural areas: a case study near Taihu Lake. *Environmental Management*.

[9] Prosdocimi M., Cerdà A., Tarolli P. (2016). Soil water erosion on Mediterranean vineyards: a review. *Catena*.

[10] Zhang T., Yang Y., Ni J., Xie D. (2019). Adoption behavior of cleaner production techniques to control agricultural non-point source pollution: a case study in the Three Gorges Reservoir Area. *Journal of Cleaner Production*.

[11] Jiang S., Qiu S., Zhou H., Chen M. (2019). Can fintech development curb agricultural nonpoint source pollution?. *International Journal of Environmental Research and Public Health*.

[12] Lu H., Xie H. (2018). Impact of changes in labor resources and transfers of land use rights on agricultural non-point source pollution in Jiangsu Province, China. *Journal of Environmental Management*.

[13] Jun H., Xiang H. (2011). Development of circular economy is a fundamental way to achieve agriculture sustainable development in China. *Energy Procedia*.

[14] Lu Y., Song S., Wang R. (2015). Impacts of soil and water pollution on food safety and health risks in China. *Environment International*.

[15] Li T., Bai F., Han P., Zhang Y. (2016). Non-point source pollutant load variation in rapid urbanization areas by remote sensing, Gis and the L-THIA model: a case in Bao’an District, Shenzhen, China. *Environmental Management*.

[16] Lou H., Yang S., Hao F. (2019). Evolution and driving forces of non-point source pollution in a developing megacity: beijing as a long-term case study. *Polish Journal of Environmental Studies*.

[17] Liu Z., Lang L., Li L., Zhao Y., Shi L. (2021). Evolutionary game analysis on the recycling strategy of household medical device enterprises under government dynamic rewards and punishments. *Mathematical Biosciences and Engineering: MBE*.

The article "Research on the Relationship between Urban Agricultural Nonpoint Source Pollution and Rural Residents' Income Growth" was published in 2022. Journal: J Environ Public Health.

[18] Liu Z., Guo H., Zhao Y. (2022). Optimal pricing decision of composite service offered by network providers in E-commerce environment. *Electronic Commerce Research*.

[19] Jiang Z. y., Hu Y. (2021). Coupling and coordination between new urbanization and agricultural modernization in Central China. *Journal of Natural Resources*.

[20] Kirby C. K., Specht K., Fox-Kämper R. (2021). Differences in motivations and social impacts across urban agriculture types: case studies in Europe and the US. *Landscape and Urban Planning*.

[21] Liu Z., Qian Q., Hu B. (2022). Government regulation to promote coordinated emission reduction among enterprises in the green supply chain based on evolutionary game analysis. *Resources, Conservation and Recycling*.

[22] Grossman G. M., Krueger A. B. (1991). *Environmental Impacts of a North American Free Trade Agreement*.

[23] Grossman G. M., Krueger A. B. (1995). Economic growth and the environment. *Quarterly Journal of Economics*.

[24] Acaravci A., Ozturk I. (2010). On the relationship between energy consumption, CO2 emissions and economic growth in Europe. *Energy*.

[25] Jiang L., Wang X. J. (2019). EKC hypothesis verification between rural environmental quality and agricultural economic growth in China——an empirical analysis based on panel data of 31 provinces. *Issues in Agricultural Economy*.

[26] Zhang H., Yu Y., Hu H. (2011). Economy growth and agricultural non-point source pollution: an empirical analysis: based on provincial panel data (1990-2007). *Energy Procedia*.

[27] Managi S. (2006). Are there increasing returns to pollution abatement? Empirical analytics of the Environmental Kuznets Curve in pesticides. *Ecological Economics*.

[28] Lin J. B., Wang Y. J., Fan X. G. (2021). Research on economic driving characteristics of agricultural non-point source pollution in Ningxia. *Journal of Arid Land Resources & Environment*.

[29] Liu Y., Mabee W., Zhang H. (2021). Conserving fertilizer in China’s rural-agricultural development: the reversal shifts and the county-specific EKC evidence from Hubei. *Cleaner Environmental Systems*.

[30] Yang J., Li J. (2020). Research on the relationship between agricultural economic growth, agricultural structure, and agricultural non-point source pollution in Fujian Province. *Chinese Journal of Eco-Agriculture*.

[31] Shi K. H., Shang J. (2021). Evolution track, effect evaluation and optimization suggestions of agricultural non-point source pollution control policies. *Reform*.

[32] Zhang L., An Y. (2018). The government capacity on industrial pollution management in Shanxi province: a response impulse analysis. *Journal of Environmental Management*.

The article "Research on the Relationship between Urban Agricultural Nonpoint Source Pollution and Rural Residents' Income Growth" was published in 2022. Journal: J Environ Public Health.

[33] Chen X. W. (2002). Environment and China’s rural development. *Management World*.

[34] Min J. S., Kong X. Z. (2016). Research development of agricultural non-point source pollution in China. *Journal of Huazhong Agricultural University: Social Sciences Edition*.

[35] Ge J. H., Zhou S. D. (2011). Analysis of the economic influence factors of agricultural non-point source pollution. *Chinese Rural Economy*.

